# Thermography as an Economical Alternative Modality to Mammography for Early Detection of Breast Cancer

**DOI:** 10.1155/2021/5543101

**Published:** 2021-07-31

**Authors:** Asim Ali Khan, Ajat Shatru Arora

**Affiliations:** Department of Electrical and Instrumentation, Sant Longowal Institute of Engineering and Technology, Longowal 148106, India

## Abstract

Breast cancer has become a menacing form of cancer among women accounting for 11.6% of total deaths of 9.6 million due to all types of cancer every year all over the world. Early detection increases chances of survival and reduces the cost of treatment as well. Screening modalities such as mammography or thermography are used to detect cancer early; thus, several lives can be saved with timely treatment. But, there are interpretational failures on the part of the radiologists to read the mammograms or thermograms and also there are interobservational and intraobservational differences between them. So, the degree of variations among the different radiologists in the interpretation of results is very high resulting in false positives and false negatives. The double reading can reduce the human errors involved in the interpretation of mammograms. But, the limited number of medical professionals in developing or underdeveloped countries puts a limitation on this remedial way. So, a computer-aided system (CAD) is proposed to detect the benign cases from the abnormal cases that can result in automatic detection of breast cancer or can provide a double reading in the case of nonavailability of the trained medical professionals in developing economies. The generally accepted screening modality is mammography for the early detection of cancer. But thermography has been tried for early detection of breast cancer in recent times. The high metabolic activity of the cancer cells results in an early change in the temperature profile of the region. This shows asymmetry between normal and cancerous breast which can be detected using different techniques. Thus, this work is focussed on the use of thermography in the early detection of breast cancer. An experimental study is conducted to find the results of classification accuracy to compare the efficacy of thermography and mammography in classifying the normal from abnormal ones and further abnormal ones into benign and malignant cases. Thermography is found to have classification accuracy almost at par with mammography for classifying the cancerous breasts from healthy ones with classification accuracies of thermography and mammography being 96.57% and 98.11%, respectively. Thermography is found to have much better accuracy in identifying benign cases from the malignant ones with the classification accuracy of 92.70% as compared to 82.05% with mammography. This will result in the early detection of cancer. The advantage of being portable and inexpensive makes thermography an attractive modality to be used in economically backward rural areas where mammography is not practically possible.

## 1. Introduction

Cancer is an uncontrolled growth of cells in any part of the body. The cells which grow in an uncontrolled manner forming abnormal cells are called cancerous cells. In some cases, cancer is confined to a particular part of the body and sometimes these cells can move to different parts of the body through the lymphatic system. The spread of these cells to other areas of the body is known as metastasis. Cancer formed in the cells of the breasts is called breast cancer. It is the most commonly occurring cancer among women. Though more common in women, it can develop in both men and women. The significant research funding results in the early detection and treatment of breast cancer. With all these advancements, deaths rates associated with this cancer are declining and survival rates have increased substantially. The main contributing factors are earlier detection and a better understanding of this type of cancer.

The most significant factor for the treatment of breast cancer is its early detection. Since the primary tumour usually does not generate any notable symptoms, the early detection of cancer should rely on performing tests in a large nonsymptomatic population. These tests are termed cancer screening tests. These are generally performed only on a limited population with greater cancer predisposition. Cancer screening is usually performed using imaging methods such as mammography, ultrasound, MRI, and thermography. Mammography is a commonly used modality to detect cancer at an early stage.

Thermography screens for breast cancer by detecting physiological changes in breast tissue, rather than anatomical ones. Specifically, thermography detects changes in heat and blood flow that are indicative of tumour growth. Once a tumour reaches a certain size, it starts generating its own blood supply in a process called angiogenesis. This, in turn, generates heat, which is detectable with thermography.

Although a mammogram can only detect the tumour that has been growing for several years, thermography can sometimes detect abnormal cell activity much earlier. If a tumour is detected early with thermography, it can often be treated without invasive surgery. So, breast cancer is detected with both mammography and thermography for the comparison purpose for the early detection of cancer. The results are compared with their relative advantages and disadvantages.

## 2. Literature Review

There are a number of research works on breast cancer detection using thermography in recent times. Gogoi et al. [1] used the statistical features, to detect abnormal breasts from normal ones in thermograms, while most of the works used the statistical features of thermograms for finding the asymmetry between the two breasts. In this paper, the Gabor features are used to capture the textural differences between the two asymmetric breasts. In [2], the feature subspaces are constructed from balanced data subsets to train different classifiers on different subspaces for the classification of thermograms. Wakankar et al. in [3] described the technique for extracting the region of interest, segmentation, and different temperature distributions among the two breasts that is used to analyse the asymmetry of the breasts. In [4], a smart system is used to make accurate and faster detection of breast cancer using thermography. An automatic method is proposed employing many image-processing techniques such as thresholding, clustering, edge detection, and refinement, for the segmentation of the thermograms [5]. Horizontal edge detection followed by Otsu's thresholding and morphological operation is used in this paper to separate the left and right breasts with good results. The thermography has been evaluated to explore the feasibility of using it as an auxiliary exam for the detection of breast cancer. The different classifiers such as Bayes Network and multiperceptron network are used in this paper [6]. Breast cancer detection from thermographic breast images using four deep learning networks has been implemented [7].

There are also a number of research works on breast cancer detection using mammography available in the literature. A number of image enhancement techniques are described in [8]. Duraisamy and Emperumal in [9] used a Chan-Vese level set to trace the contours of the mammograms for segmentation. A scalable approach for retrieval and diagnosis of mammographic masses is proposed by Jiang et al. in [10]. Rangaraj et al. in [11] applied a region-based method of image edge profile acutance to characterize the variation in density of a region of interest (ROI). The most commonly used texture features in mammographic images are described in [12] by Haralick et al. A number of methods of classifications, both unsupervised and supervised, are used to classify the mammograms. In [13], Li et al. used the K-means which works by specifying the number K of clusters expected and calculating the intraclass distance and reattached cluster centres according to distance values. The support vector machine is used as a classifier with RBF kernel in this paper for the classification with the results among the best in the literature. In [14], the microcalcifications are classified using different state-of-the-art machine-learning methods. An active contour method based on a reformed combined local and global fitted function is used for the segmentation of the mammograms [15]. A CAD method is designed using feature fusion with convolutional neural network (CNN) deep features [16]. The similarity between neighbouring regions of masses is detected by using two new features, to capture global similarity at different scales. In addition, uniform local binary patterns are computed to increase the classification accuracy by combining with these features [17].

## 3. Methodology

The thermal images with ground truths for cancerous and noncancerous breasts are acquired online from Database for Mastology Research Database [18]. The DMR-IR contains IR images and clinical data obtained from patients of the Hospital Universitário Antônio Pedro (HUAP) of the Fluminense Federal University, Brazil.

The procedure of extracting the region of interest (ROI) is shown in Figure 1. The unwanted area of the thermogram is manually cropped before converting it into the grayscale image. Here, an algorithm has been proposed which not only removes the background area but also extracts the left and right breast areas by using horizontal edge detection [19]. Horizontal edge detection is done by following Otsu's thresholding and morphological operation.

These steps are summarised in the flowchart for extraction of the region of interest (ROI) and segmentation as shown in Figure 2.

In a normal breast thermogram, the temperature pattern of both the left and right breasts is closely symmetrical. A breast tumour may result in temperature changes between the two breasts. Thus, an asymmetry in the thermal pattern of both breasts may signify breast pathology. For identifying a minute difference in the temperature pattern of both breasts, asymmetry analysis of both breasts is done using the textural differences between the two breasts which is captured by the Gabor texture features.

The texture features are described for texture representation and discrimination. Bovik et al. used a technique for finding filters by using texture power spectrum features [20]. Jain and Farrokhnia proposed a dyadic Gabor filter bank to analyse the spatial-frequency domain [21]. Many research papers reported Gabor features to be effective in extracting the textural description [22–24]. A multiresolution feature extraction approach for characterizing the textural properties is used. In this pattern, textural properties are characterized at various scales and orientations for an improved separability between the different extracted features. It can be considered as a Gaussian modulated sinusoid having multiresolution decomposition in the spatial and spatial-frequency domain. The real impulse response of a 2D sinusoidal plane wave is given as

(1) $$\begin{array}{c} g\left(x,y\right)=\frac{1}{2\pi \rho_{x}\rho_{y}}\left\{-\frac{1}{2}\left[\frac{x^{2}}{\rho_{x}^{2}}+\frac{y^{2}}{\rho_{y}^{2}}\right]\right\}, \end{array}$$

where *x* = cos*θ* + sin*θ* and *y* = −*x*sin*θ* + *y*cos*θ*.

The Gabor filter in the corresponding spatial-frequency domain would be represented as two symmetrically spaced Gaussian functions as follows:

(2) $$\begin{array}{c} g\left(x,y\right)=\exp\left\{-2\pi^{2}\left|{\left(u-f\right)}^{2}\sigma_{x}^{2}+v\sigma_{y}^{2}\right|\right\}+\exp\left\{\left|{\left(u-f\right)}^{2}\sigma_{x}^{2}+v\sigma_{y}^{2}\right|\right\}. \end{array}$$

The Gaussian envelope unknowns *σ*_*x*_ and *σ*_*y*_ can be determined as in equation (3), after setting frequency cutoff to −6 db and the frequency and orientation bandwidths to constant values matching psycho visual data. This was inspired by experiments showing that the frequency bandwidth of simple cells in the visual cortex is roughly one octave. For this work, a circular Gaussian function was chosen by setting *σ*_*x*_ = *σ*_*y*_ to have an equal spatial coverage in all directions and a 45° orientation bandwidth:

(3) $$\begin{array}{c} {ο}_{x}=\frac{\sqrt{\ln\;2}\left(2^{B+1}\right)}{\sqrt{2}\pi \left(2^{n}-1\right)}{ο}_{y}=\frac{\sqrt{\ln\;2}}{\sqrt{2}\pi f\;\tan\left(B_{0}/2\right)}.\; \end{array}$$

The careful setting of the filter characteristics would result in proper capture of the texture information and reduce the effect of aliasing. This is achieved by correctly selecting the filter position (*f*_0_, *θ*) and bandwidth (*σ*_*x*_, *σ*_*y*_) and making sure that the central frequencies of channel filters lie close to characteristic texture frequencies to prevent the filter response from falling off too rapidly. From each of the images used in this work which have a size of 1024 × 1024, the mean was first subtracted to reduce the filter's sensitivity to texture with constant variation; then, four radial frequencies of 0.25, 0.176, 0.125, and 0.088 with five orientations of 0°, 36°, 72°, 108°, and 144° were adopted, giving a total of 20 filters. The orientations (*O*) and frequencies (*F*) for a bank are calculated using the following two equations, respectively:

(4) $$\begin{array}{c} O=\frac{\left(j-1\right)\pi }{V},\;\text{where }j=1\text{ to }5, \end{array}$$

(5) $$\begin{array}{c} F=\frac{f_{\max}}{\sqrt{2^{i-1}}},\;\text{where }j=1\text{ to }5. \end{array}$$

Applying a set of filter banks resembles the operation of a wavelet transforming an image at selected spatial frequencies. In a way, the Gaussian function is modulated and translated for the generation of the Gabor basis functions, in analogy to the scaling and translation of the mother wavelet and scaling function for wavelet basis generation. However, the Gabor function is considered an admissible wavelet, namely, the basis produced by the Gabor function. It is a nonorthogonal wavelet resulting in redundant decompositions. Also, depending on the size of the processed image, the number of required radial frequencies for positioning the centers of the Gabor filters banks needs to be specified prior to processing, which is similar to choosing the number of decomposition levels for the wavelet packets.

The classical method for extraction of Gabor filter texture signature is the energy *E*_*k*_, *k* = 1, 2 as in the following equation, where *M* and *N* are the sizes of the subband intensity:

(6) $$\begin{array}{c} E_{k}=\sum_{x=0}^{M-1}\sum_{y=0}^{N-1}{\left[I\left(x,y\right)\right]}^{k}. \end{array}$$

After the banks have been constructed, each segmented image is convolved with the filter bank having five orientations and four frequency shifts, which gives a total of 20 features (absolute mean or energy). The Gabor features for the left and right breasts are subtracted to find the asymmetry between the two breasts.

The average of the Gabor features plotted for normal and abnormal thermograms is shown in Figure 3.

The classification of the thermograms into healthy and cancerous, and benign and malignant classes is done using the SVM [25]. The parameters used in the SVM classifier are given in Table 1.

In this case, a straight line cannot separate the data points; then, the kernel trick is used to separate such data. The basic idea behind the kernel trick is to add another dimension. The RBF kernel is used in this paper. The *C* parameter denotes a penalty for each misclassified data point. If *c* is small, the penalty for misclassified points is low so a decision boundary with a large margin is chosen at the expense of a greater number of misclassifications. If *c* is large, SVM tries to minimize the number of misclassified examples due to high penalty which results in a decision boundary with a smaller margin.

The gamma parameter is used if the RBF kernel is used. The gamma parameter of RBF controls the distance of influence of a single training point. The low values of gamma indicate a large similarity radius which results in more points being grouped together. For high values of gamma, the points need to be very close to each other in order to be considered in the same group or class.

The results of the classification of normal/abnormal thermograms using Gabor features and SVM classifier are shown in Table 2.

The thermography achieved an average accuracy of 96.57% with maximum accuracy of 100%. This better accuracy is attributed to the subtracted features instead of all features given to the classifier. The sensitivity of 100% means no missed cancerous case that is an important characteristic of the computer-aided diagnosis system in medical applications. As the missed cases can result in the death of the patient. The specificity is also reasonably good, that is, less number of false-positive cases.

The classification accuracy achieved in this paper is compared with the existing literature available and displayed in Table 3. It is found to be the highest among all the existing works.

Further, the cancerous thermograms are classified into benign and malignant ones using the difference of Gabor features of the left and right breasts and the SVM classifier. The results of the classification of benign/malignant thermograms using Gabor features and SVM classifier are shown in Table 4.

The average accuracy obtained with this approach is 92.70% with maximum accuracy of 100%. The accuracy is found to be very encouraging in the early detection of cancer as the benign cases can be traced at an early stage.

## 4. Comparison of Thermography with Mammography for Breast Cancer Detection

The quantitative comparison of thermography and mammography for early detection of cancer is done in this paper. For this purpose, the mammographic images are taken from the mammographic image analysis society (MIAS). There are a total of 322 digitized mammograms of both breasts of 161 women [26]. The standard size of every image is 1024 × 1024.

The required preprocessing steps such as artefact removal, pectoral muscle removal, and denoising using Gaussian difference are performed on the mammograms [26] and the region of interest is extracted using an automatic cropping algorithm. The segmentation of the cropped image is done using the Level Set Method. The active contour based models are based on the idea of creating a curve subjected to limits from the image to identify the objects in that image. For example, a curve is evolved around the object to be identified, the curve moves toward its interior normal and will stop on the boundary of the object [27]. Thapaliya et al. in [28] proposed the Level Set Method for the segmentation.

The texture based features are extracted using Haralick's features. The texture analysis with the use of cooccurrence probabilities using gray level cooccurrence matrix (GLCM) was introduced by Haralick et al. in [12]. The GLCM is a 2D histogram of gray levels for two pixels at a fixed spatial distance. GLCM of an image is found using radius *d* and orientation *θ*. The numbers of rows and columns in the matrix are decided by the number of gray levels *G*, in the given image. The classification is performed using an ensemble classifier to classify the mammograms into normal, benign, and malignant cases. An ensemble classifier is the combination of classifiers in which the decisions of the classifiers are computed and combined by some fixed algorithm. Very active research is in progress to find the best methods to combine the outputs of the individual classifiers for an efficient ensemble classifier. It has been reported in a number of studies and concluded in this work also that the ensemble classifiers' performance is better than the individual classifiers that constitute the ensemble classifier.

The results of the classification of mammograms into normal/abnormal and abnormal into benign and malignant are presented in Tables 5 and 6, respectively.

Then, the masses are classified into normal and abnormal masses using ensemble classifiers with an overall accuracy of 98.11%.

The accuracy obtained is 82.05% for the classification of benign and malignant mammograms. The classification accuracy in the case of masses/nonmasses is much higher than in the case of benign and malignant cases. This may be due to the very small textural differences between the benign and malignant mammograms where the textural differences are substantial in the case of normal and abnormal mammograms. As the false positives in this classification can result in an unnecessary biopsy, the false negative will miss out the malignant cases. This is one of the fallouts of mammographic imaging that the classification accuracy is quite less in benign/malignant classification.

## 5. Discussion

Mammograms are classified into normal and cancerous ones using the SVM classifiers with an average accuracy of 98.11% as compared to the average accuracy of 96.57% achieved with thermography. The performances of the two modalities are almost the same. In addition, thermography has a sensitivity of 100% which ensures no missed case of breast cancer that can be otherwise life-threatening. The cost of misclassification is more in false negatives as compared to false positives. As in the case of thermography, there are no false negatives, so the cost of misclassification is quite less with no cancerous patient being untreated.

In classifying the malignant and benign cases in the cancerous cases, thermography is far ahead in classification accuracy in comparison with mammography with an accuracy of 92.70% as compared to 82.01% of mammography. The thermography in this case also has a sensitivity of 100%, so all malignant cases are identified. This ensures that no biopsy is recommended for benign cases, avoiding the unnecessary cost and anxiety of the patient. The early detection of benign cases with thermography can save several lives. So, thermography is found to give much superior performance in classifying the benign/malignant case while having an additional advantage of achieving a 100% sensitivity in classification of both normal/abnormal and benign/malignant cases.

## 6. Conclusion

The accuracy achieved in detecting breast cancer in mammography screening is 98.11% which is slightly higher than the accuracy of 96.57% achieved using thermography. This suggests that thermography has come a long way to match the accuracy of the modality of mammography. The sensitivity obtained with thermography is 100% which suggests no false negatives in the case of the thermography screening tool. The finding in this work is the ability of the thermography to identify the benign cases from the malignant with a reasonably good accuracy of 92.70%. This classification is very poor, that is, 82.05% in the case of mammography. So, the technique of thermography is very useful in this aspect of avoiding unnecessary biopsies in the case of benign breast cancer and identifying the early cases of breast cancers. The foremost is the changes in breasts due to angiogenesis come much earlier as compared to anatomical changes detected by mammography. The successful identification of the malignant cases gives it an edge over the mammography.

With this very encouraging accuracy achieved and inbuilt advantages of low cost, portability, and painless procedure of the thermography, it can be a viable alternative to the presently used mammography. This is particularly useful in rural and economically backward areas. A computer-aided design (CAD) system can be designed using thermography for automatic detection of breast cancer or can be used for second reading.

This has a very significant impact in developing countries in which there is less availability of medical personnel. The low cost involved in the thermography will help the limited-resource communities in providing the screening modality for the early detection of breast cancer. The early detection of cancer will lessen the load on the limited medical infrastructure of underdeveloped communities. The portability of the thermography makes its access possible in rural areas where mammography is not possible.

By further advancements in thermal camera technology and more efficient computational techniques, thermography will become a more potent method for early detection of breast cancer with the above-mentioned findings and the listed advantages.

## Figures and Tables

**Figure 1:** Region of interest extraction.

**Figure 2:** Flowchart for extracting ROI and segmentation.

**Figure 3:** Average of Gabor features of normal and abnormal thermograms.

**Table 1:** SVM parameters used in the classification.

Kernel	*C* parameter	Gamma
Radial basis function (RBF)	2	2

**Table 2:** Results of classification of normal/abnormal thermograms using Gabor features and SVM classifier.

Iterations	Sensitivity	Specificity	Accuracy (%)	Error rate (%)	Precision	MCC	F-score
1	1	0.8235	91.18	8.82	0.85	0.8235	0.9189
2	1	0.9412	97.06	2.94	0.9444	0.9412	0.9712
3	1	0.9412	97.06	2.94	0.9444	0.9412	0.9712
4	1	1	100	0	1	1	1
5	1	0.8824	94.12	5.88	0.8947	0.8824	0.9444
6	1	1	100	0	1	1	1
Maximum	1	1	100	8.82	1	1	1
Minimum	1	0.8235	91.18	0	0.8947	0.8824	0.9189
Mean ± SD	1	0.9314	0.96.57	3.4300	0.9389	0.9314	0.9676
	±0	±0.0688	±3.4370	±3.4370	±0.0590	±0.0688	±0.0317

**Table 3:** Comparison of the proposed method of thermography and results of other research findings.

S. no.	Reference	Methodology	Database	Results (%)
1	Rangaraj et al. [11]	ANN		61.54
2	Haralick et al. [12]	Biostatistical methods and artificial neural networks (ANNs)	—	80.95
3	Li et al. [13]	ANN + RBFN		80.95
4	Wei et al. [14]	Statistical features	—	85.71
5	Niaz et al. [15]	Statistical image features	Brno University of Technology	91.09
6	Wang et al. [16]	Bayesian network		71.88
7	Rabidas et al. [17]	Image symmetry features	Brno University of Technology	90.03
8	Silva et al. [18]	SVM + RBF		90
9	Bovik et al. [20]	CNNs		92
10	Jain and Farrokhina [21]	Multilayer perception		95
11	Proposed method	Gabor features and ensemble classification	DMR (Database for Mastology Research) database	96.57

**Table 4:** Results of classification of benign/malignant cases using Gabor features and SVM classifier.

Iterations	Sensitivity	Specificity	Accuracy (%)	Error rate (%)	Precision	MCC	F-score
1	1	1	100	0	1	1	1
2	1	0.875	93.75	6.25	0.8889	0.875	0.9412
3	1	0.75	87.50	0.125	0.8	0.75	0.889
4	1	0.75	87.50	0.125	0.8	0.75	0.889
5	1	0.875	93.75	6.25	0.8889	0.875	0.9412
6	1	0.875	93.75	6.25	0.8889	0.875	0.9412
Maximum	1	1	100	6.25	1	1	1
Minimum	1	0.75	87.50	0	0.8	0.75	0.889
Mean ± SD	1	0.8542	92.7083	3.1667	0.8778	0.8542	0.9336
	±0	±0.0941	±4.7048	±3.3779	±0.0740	±0.0941	±0.0414

**Table 5:** Ensemble classification validation measures for masses/nonmasses using GLCM features.

Iterations	1	2	3	4	5	6	7	Mean ± SD
Majority Voting	0.9877	0.9789	0.9822	0.9789	0.9733	0.9877	0.9789	0.9811 ± 0.005
Maximum	0.9732	0.9732	0.9732	0.9732	0.9732	0.9732	0.9732	0.9618 ± 0.108
Sum	0.9877	0.9789	0.9822	0.9789	0.9733	0.9877	0.9789	0.9811 ± 0.005
Minimum	0.9698	0.9610	0.9643	0.9559	0.9425	0.9602	0.9469	0.9572 ± 0.010
Average	0.9877	0.9789	0.9822	0.9789	0.9733	0.9877	0.9789	0.9811 ± 0.005
Product	0.9798	0.9510	0.9643	0.9569	0.9425	0.9612	0.9469	0.9575 ± 0.0125
Bayes	0.9698	0.9510	0.9822	0.9704	0.9376	0.9644	0.9469	0.9603 ± 0.016
Decision Template	0.9877	0.9789	0.9822	0.9789	0.9733	0.9877	0.9789	0.9811 ± 0.005
Dempster–Shafer	0.9877	0.9789	0.9822	0.9789	0.9733	0.9877	0.9789	0.9811 ± 0.005

**Table 6:** Classification of benign and malignant using different combining methods of ensemble classifiers [29].

Iterations	1	2	3	4	5	6	7	Mean ± SD
Majority Voting	0.8573	0.7800	0.8469	0.8377	0.7244	0.7429	0.8099	0.7999 ± 0.052
Maximum	0.7609	0.6558	0.7614	0.7892	0.6885	0.7636	0.7810	0.7429 ± 0.050
Sum	0.8573	0.7800	0.8469	0.8377	0.7244	0.7429	0.8099	0.7999 ± 0.052
Minimum	0.7707	0.6852	0.7233	0.7892	0.6797	0.7832	0.7712	0.7432 ± 0.046
Average	0.8573	0.7800	0.8469	0.8377	0.7244	0.7429	0.8099	0.7999 ± 0.052
Product	0.7707	0.6852	0.7233	0.7892	0.6797	0.7832	0.7712	0.7432 ± 0.046
Bayes	0.8382	0.8279	0.7794	0.7887	0.7914	0.7914	0.7903	0.8010 ± 0.022
Decision Template	00.8671	0.8094	0.8660	0.8377	0.7614	0.7919	0.8099	0.8205 ± 0.038
Dempster–Shafer	0.8573	0.8094	0.8660	0.8377	0.7712	0.7919	0.8099	0.8205 ± 0.034

## Data Availability

A research organization in the United Kingdom, Mammographic Image Analysis Society (MIAS), provides a database of digital mammograms online at http://www.mammoimage.org/databases/. The thermal images for cancerous and noncancerous breasts are acquired online from the Database for Mastology Research at http://visual.ic.uff.br/en/proeng/thiagoelias/.
